The article "Stress-Relieving Video Game and Its Effects: A POMS Case Study" was retracted in 2023. Reasons: unreliable results or conclusions; lack of ethics approval or compliance; missing or withdrawn patient consent; concerns about the data.

# Stress-Relieving Video Game and Its Effects: A POMS Case Study

**DOI:** 10.1155/2022/4239536

**Published:** 2022-04-20

**Authors:** Abdullah Ajmal, Hamza Aldabbas, Rashid Amin, Sundas Ibrar, Bader Alouffi, Mehdi Gheisari

**Affiliations:** ^1^Department of Computer Science, University of Engineering and Technology, Taxila, Pakistan; ^2^Prince Abdullah Bin Ghazi Faculty of Information and Communication Technology, Al-Balqa Applied University, Al-Salt, Jordan; ^3^Department of Computer Science, College of Computers and Information Technology, Taif University, P.O. Box 11099, Taif 21944, Saudi Arabia; ^4^Department of Computer Science and Technology, Harbin Institute of Technology, Shenzhen, China; ^5^Department of Computer Science, Islamic Azad University, Tehran, Iran

## Abstract

Stress is the response or a change in our bodies to environmental factors like challenges or demands that are physical and emotional. The main cause of stress is illnesses and it is gaining more interest, a hot topic for many researchers. Stress can be brought about by a wide range of normal life occasions that are hard to avoid. Stress generally refers to two things: first, the psychological perception of pressure and the body's response to it. On the other hand, it involves multiple systems, from metabolism to muscles to memory. Many methods and tools are being developed to reduce stress in humans. Stress can be a short-term issue or a long-term problem, depending on what changes in your life. The emphasis of this article is to reduce the effects of stress by developing a stress-releasing game and verifying its results through the Profile of Mood States (POMS) and POMS-2 survey. Games are associated with stress levels; hence, parameters like sounds, visuals, and colors associated with reducing stress are used to develop a game for the stress reduction in the players. The survey research aims to determine that the purpose-built game will affect the player's stress level using a reliable psychological survey paper. The survey collected a variety of information from its participants over six months. Different aspects of a person's psychology and reactions are recorded in this scenario by calculating the mean, standard deviation, degree of freedom, zero-error, and probability-value%. The POMS and POMS-2 results are obtained from the custom-built game, and these are found to be effective in reducing stress.

## 1. Introduction

Profile of Mood States (POMS) is a recognized test first formulated by McNair et al. (1971) [1]. The survey includes 65 questions to represent the mood state of the participant. The POMS is a mechanism for measuring mood. The POMS and POMS-2 test cannot be used in clinical psychology, psychotherapy, and sports science. The POMS and POMS-2 represent the exclusively appropriate mechanism to measure mood-related symptoms properly. In addition, the results point to exact indications related to the place of work-related well-being. The previous revision points out the psychometric results for the POMS and POMS-2 tests. Its multidimensionality is beneficial for research. POMS and its 2^nd^ edition are ready to provide data to evaluate workplace-related stresses and do not need much effort [2]. POMS classify anger as an emotional situation that ranges from minor impatience feelings until the anger is linked to stimuli from the autonomous nervous system. POMS and POMS-2 define mental disturbance as confusion, insecurity of interest and emotions, depression reduction, and deprived self-image. The fatigue issue clarifies the sense of physical, mental tiredness, and tension factor or feelings up to the time of worry, anxiety, vigor issue, as differentiated by enthusiasm, temper, and physical energy. COVID-19 has caused significant distress around the globe. It is not limited to adults only, but stress is increasingly affecting children of all age groups. Countries worldwide implemented strict precautions on their citizens in an attempt to control the spread. Most stressing is quarantine. The survey is evaluated and the selection of the psychoanalysis component will depend on the purpose of assessing everyone at some viewpoints with dissatisfaction. There is more than one cause, which includes various circumstances such as losing a loved one, work, and even the weather, which causes a damp and troubling condition known as regular full of feeling clutter disorders. The Profile of Mood States 2^nd^ edition was published in 2012 by the Multi-Health System (MHS) to assess transient feelings and mood among individuals aged 13 years and above. It was designed to cover the age between 13 and 17 years old and adults aged 18 years and above to measure their effective moods and emotions. To enhance their mood, humans will generally discover social embrace or do exercise; these activities can be different for everyone. According to one estimate, 4.4% of the global population suffer from stress and 3.6% from anxiety disorder, whereas depression is more common, at 7.5%, with anxiety being the sixth-highest disorder, and both are estimated to increase. Hence, therapies like cognitive behavioral therapy (CBT) are essential treatments to investigate treatment [3]; those who do not face the disorder longer respond to either pharmacological or psychological interventions, which are frequently encouraged as fast remedies for anxiety and depression. Such approaches provide more options to consider client preferences, treatment accessibility, charge for enlarging devotion, and suitability.

The article "Stress-Relieving Video Game and Its Effects: A POMS Case Study" was retracted in 2023. Reasons: unreliable results or conclusions; lack of ethics approval or compliance; missing or withdrawn patient consent; concerns about the data.

Other methods like digital involvement, including online, computerized apps, and serious games, ensure reducing depression and anxiety symptoms. This study was performed to observe a player's mental stress while playing a stress-releasing game specifically built to release the player's stress levels. According to the National Institute of Mental Health, about 20.9 million or 9.5% population in the USA aged 18 years or older face temperament disorders. In total, 14.8 million adults between the ages of 15 and 44 have depression concerns [4]. Moreover, 1.5% and 3.3 million of the population in the USA are affected by Dysthymic Disorder. At the beginning, the middle ages have disorder for just about 30 years (National Institute of Mental Health) [5]. Stress is usually familiar because of a person's state when too much is predictable, regarding severe pressure or strain, and when they are hardly capable of dealing with excessive and wide exterior demands. Stress is taken as ecological demand as it affects the human organism and if not resisted, it would be unsafe. Casual video games (CVG) have around 200 million players globally. The culture and ages provide a vast diversity in the electronic gaming communities online and offline playing the games on various platforms like PC and handheld cellular phones. These can be further elaborated by the Casual Games Association's 2008 report, which stated that the most opened application on Windows XP was Microsoft Solitaire. According to the 2006 JWT Intelligence report, the CVG or web games business will grow to $55 billion by 2009. The world's most stressful countries yearly are shown in Table 1, Table 2, and Table 3.

The idea of the study is to conclude that a video game may improve mood and reduce stress using appropriate measurements. CVG is related to deliberation in its effects on physiological stimulation, suspected confidence, and harm mood. The mere exemption is an augmented helpful influence intended for mood. The outcome supported the prediction that CVG can be a suitable way to reduce stress in the subjects. The results of this study evaluated the positive effects of CVG on stress levels compared to other methods like yoga and meditation. CVG induces an increase of alpha signals in the right frontal part of the brain and reduces it in the left frontal part. The rise of alpha in the left hemisphere is linked to negative behavior like depression, bad mood, and avoidance. At the same time, the increase of alpha in the right hemisphere improves the overall mood and makes a person more engaging. These relations of alpha waves in the right and left parts of the brain are discussed in [6]. The most used scale for measuring positive and negative effects on mood is the Positive and Negative Affect Schedule (PANAS). The PANAS in several languages has exposed first-rate psychometric possessions in the all-purpose clinical samples and population, including women with fibromyalgia, drug addicts, and samples of forensic nature. PANAS has not been examined on depressive and anxiety disorders and other clinical samples. Furthermore, the advent of treatments based on the Internet has expanded into a diverse range of similar scales that can be performed online, such as online surveys and feedback forms. We are conducting this survey research to eliminate stress using the POMS and POMS-2 tests [7]. Our goal is based on this survey research that will work for people's moods in a few minutes. We have to manage anxiety, stress, depression, fatigue, confusion, unhappiness, and vigor. With this test, we can keep ourselves relaxed to a great extent. Our test will significantly reduce stress. The following are the key contributions of this article:

- Evaluation of the POMS and POMS-2 survey is performed to reduce stress among those who are using purpose-built games.
- The effects of casual gaming on stress are highlighted by performing a survey in which the measurement of Total Mood Disturbance (TMD).
- The change in stress is evaluated by performing surveys and purpose-built games. The level of stress in several ways is reduced, including calculating mean, standard deviation, zero-scale, and probability-value.

The article "Stress-Relieving Video Game and Its Effects: A POMS Case Study" was retracted in 2023. Reasons: unreliable results or conclusions; lack of ethics approval or compliance; missing or withdrawn patient consent; concerns about the data.

The rest of the article is organized as follows.  Section 2 presents the literature review, and Section 3 offers the problem statement. The proposed solution is discussed in Section 4, and the results are included in Sections 5 and6 . We concluded the article in Section 7.

## 2. Literature Review

Video games are becoming popular and more interactive day by day [8]. Due to the effects of video games on mood, several neurologists are becoming more interested in them. Because of their nature, video games take part in a generous responsibility in feeling and significantly put into individual behavior and cognitive functions [9]. According to Reinecke, the contributors required by the game decrease the capability of players to think over demanding events. The physiological relaxation provided by video games differs widely between games and is not always an accurate representation of stress [10].

Reinecke's (2009) study presented an idea for the revival of stress regarding four distinct parts, including psychological disinterest, physiological relaxation, mastery experiences, and apparent control [11]. The four major aspects are used to reduce stress hypothetically to show that video games reduce stress and aid in healing. For this study, the game was intended to determine stress reduction. It builds ongoing investigation by joining physiological events to observe the probable stress-reducing effects of video gaming. According to the “Casual Games Association” (2013), over 200 million people take part in CVGworldwide [12]. The association aims to look at stress and reduce the effects of casual games compared to guided relaxation. PANAS Mood scale test and Dundee Stress State Questionnaire (DSSQ) were used for the dimensions and a stress-inducing task [13]. CVGs were always efficient as a form of stress relief and were extra productive to engage the contributors. CVGs are taken as meditation and to reduce stress. It was completed using suitable physiological measures to resolve changes in physiological stimulation and mood. In previous studies, one unique thing is to highlight different games such as ‘‘Bejeweled 2,” ‘‘Personal Zen,” ‘‘Plants vs. Zombies,” ‘‘Bubble Shooter,” “Peggle,” and “Bookworm Adventures” with their positive impacts on how these games can reduce our stress [14].

The article "Stress-Relieving Video Game and Its Effects: A POMS Case Study" was retracted in 2023. Reasons: unreliable results or conclusions; lack of ethics approval or compliance; missing or withdrawn patient consent; concerns about the data.

Additionally, when people put their all into their treatment plan, their outcomes frequently are improved, such as reduced anxiety and stress-related symptoms [15]. Previous studies use the “Rich get Richer” model to explain that the less worried individuals manage to play World of Warcraft (WoW) to improve their offline lives [16]. Encouraging amazingly pushed players more increment the stretch enduring in their lives by playing dangerously the online amusement inside which they are required protect from their offline inconveniences which for greatly focused people amplifies to some degree than soothing their enduring. It is important to investigate how in-game encounters and exercises shape mental diversion, leading to risky play among more focused individuals [17]. They pursued their participant observation ethnographic inquiry with 28 semistructured interviews, resulting in increased stress. The previous reading recognized more than 900 studies, from which duplicates were detached and leftover abstracts read. Around 21 articles were potentially relevant to the succeeding environment of our theories related to stretch and tricky online gaming. Perceived Stress Scale (PSS) is used in this survey, which defines stress as respondents' superficial intensity of control over their lives, with a higher score representing a high perceived stress [18]. Recently published articles exploring the thought of utilizing a CVG and pointing to the impacts of CVG's on the signs of uneasiness, misery, and stretch were then selected based on the consideration and prohibition criteria [19].

The article "Stress-Relieving Video Game and Its Effects: A POMS Case Study" was retracted in 2023. Reasons: unreliable results or conclusions; lack of ethics approval or compliance; missing or withdrawn patient consent; concerns about the data.

Using cardiac coherence, stress was accurately measured. Cardiac coherence improves as the rhythm of the heart is managed. The stress pilot biofeedback device was used to increase cardiac coherence (CC). Contributors were randomly assigned to appoint in amusement by violent and peaceful game for 20 minutes while cardiac reliability was recorded. Participants' emotional changes were evaluated on different survey papers for psychological analysis of mood, with the POMS test being the most successful. POMS measures six different scales: “Tension, Depression, Anger, Vigor, Fatigue, and Confusion.” POMS test inside reliability has been reported at about 90 or above. POMS test dependability lies between 68 and 74 for all factors. The previous research presented the point that CVG can be an effective means of reducing stress. In the article, purpose-built stress-reducing video gaming is analyzed using POMS and POMS-2 [20].

## 3. Problems' Statement and Proposed Solution

Stress is the body's standard reaction when changes occur, resulting in physical, enthusiastic, and mental reactions. Moreover, emotional and physical signs typically in the student population, including headaches, fatigue, sadness, anxiety, and the incapability toward control, can intensify by stress. It reveals a 58% increase in stress [21]. Stress causes the body to overflow with hormones that prepare its systems to pass up or tackle danger. Stress can control all aspects of your life, consisting of your emotions, behaviors, thinking ability, and physical health. The fundamental cause of stress in a youngster's life comes from work, exercise, companions, and family. There are two structures. The principal structure is called acute stress, which lasts for a short period. The causes of stress come with both internal and external effects. It depends on the person, but the internal effects include anxiety, irritability, and nervousness. External effects include breathing faster, sweating, muscles tensing, dry mouth, keener senses, lack of energy, headaches, and sickness. A stressed person tends to have trouble paying attention and have trouble recalling facts. Each day stress builds up in a teenager's life, which can be negative as this carries into their adulthood. We are conducting this survey research to eliminate stress because of using the POMS and POMS-2 tests. POMS is a psychological test prepared by McNair et al. (1971)[22]. The POMS test is considered to measure fixed psychological traits. The survey consists of 65 statements to explain the feelings of people. The POMS test can be reviewed swiftly due to the ease of the experiment. A long time ago, the POMS test had six different extents of mood swings. The measurement of the POMS test provides a fast, cheap method of reviewing transient, changeable active mood states. POMS test is an ideal mechanism for measuring and monitoring moods. It allows fast estimation of “transient, fluctuating feelings, and enduring effect states.” The Profile of Mood States 2nd Edition–Adult (POMS 2–A) is a self-report assessment of mood that is adaptable to capturing transient and fluctuating feelings or relatively enduring states in adults aged 18+ years. When used in combination with other information, results from the POMS 2–A can help to better understand an individual and guide intervention decisions.

The article "Stress-Relieving Video Game and Its Effects: A POMS Case Study" was retracted in 2023. Reasons: unreliable results or conclusions; lack of ethics approval or compliance; missing or withdrawn patient consent; concerns about the data.

There are several ways to reduce stress by doing physical exercise as it is a great way to alleviate stress. Exercise allows us to get up and go and lowers blood pressure while increasing our ability to deal with stress. Therapies can also reduce the level of stress, including yoga, meditation, and cognitive behavioral therapy (CBT). POMS and POMS-2 are effective tests because of the simplicity and ease of participant understanding. Both are considered as short tools through good quality psychometric properties that can be performed on healthy and unhealthy people. Our goal is based on this survey research on people's mood management. Using the POMS and its 2^nd^ Edition of POMS, we have to manage anxiety, stress, depression, fatigue, confusion, unhappiness, and vigor.

Figure 1 shows the methodology of the POMS test where TMD is calculated in a controlled environment and then once after the target exercise has been performed.

## 4. Methodology

For the survey, a game was developed using Unity Engine Development Tool using C# language. The assets used in-game were designed and developed by the author keeping in mind the colors, textures, and lightning that are typically used for releasing stress. The game does not have any hardness levels as it is not a competitive game and focuses on a stress-free environment throughout the game, but it does have three different scenarios of infinite maps (never-ending maps like subway surfer).

For analysis, POMS and POMS-2 survey was performed; a rating scale of psychological nature was used to calculate different states of mood. It is an authenticated test formulated by McNair in the McNair et al. (1971) [23]. POMS-2 is developed by MHS. The survey consists of 60–65 questions that evaluate a person's mood. POMS and its 2^nd^ edition require the participant to choose the best possible statement about the state mood they are feeling at that moment. POMS has a pool of 65 different questions divided into six main categories (“tension, depression, anger, vigor, fatigue, and confusion”) and is a “Last Week” or “Right Now” management. Internal dependability was reported as 90 or above. For all variables, test reliability is recorded among 68 and 74 [24].

The article "Stress-Relieving Video Game and Its Effects: A POMS Case Study" was retracted in 2023. Reasons: unreliable results or conclusions; lack of ethics approval or compliance; missing or withdrawn patient consent; concerns about the data.

Figure 2 shows the purpose-built game played for this survey to evaluate the participants' stress levels before and after the gameplay. POMS and its 2^nd^ edition were used previously for four main research areas: controlled drug evaluation, psychoanalysis, and therapy, different responses to affecting conditions, and simultaneous validity coefficients and other POMS test show a relationship. For each of the 65 questions, there are five options given as “Not at all” for 1 and up to “Extremely” for 5. The participant will select the option on the mood he/she is experiencing at that moment. The TDM score of each test is calculated by adding up the categories of “tension, depression, fatigue, confusion, and anger” and then subtracting the total score of the vigor. The tension, depression, fatigue, confusion, and anger categories are weighted as negative in the TDM score, while the vigor is weighted positively. TMD of the POMS and POMS-2 provides an accurate description of the participant's mood. The POMS test and its 2^nd^ edition have always been reported independently for the five or six factors, which is also followed in research. POMS and POMS-2 also provide reliable results on the levels of state of anxiety in the participants. Many modifications have been made in POMS and POMS-2 for different environment settings and world regions and provide fewer time-consuming surveys.

## 5. Development and Properties of Game

### 5.1. Participants

People between 18 and 30 years old and adults are selected for this survey; the participant's mean age was 23 years.

### 5.2. Administration

For 5 to 10 minutes, the paper-and-pencil self-report measure requires accomplishment users. The psychometric assessment's purpose is to reduce stress. People filled the survey papers before and after accordingly to reduce the level of stress.

### 5.3. Reliability and Validity

Multiple studies examining several patient groups and the study investigating the structure of the level established significant support for the majority of the POMS seven variables and the subscale fatigue-inertia was established to have exclusive honesty.

Figure 3 defines the psychological effects on the human being, both physically and mentally. These show psychological effects on tension, anger, fatigue, confusion, and vigor are the main building block that causes stress.

The article "Stress-Relieving Video Game and Its Effects: A POMS Case Study" was retracted in 2023. Reasons: unreliable results or conclusions; lack of ethics approval or compliance; missing or withdrawn patient consent; concerns about the data.

### 5.4. Scoring

It involves respondents pointing out that every point describes their frame of mind in an overload before and after using a 5-point scale ranging from “Not at all” to “Extremely.” POMS is obtainable in an immediate scoring format, in which the participant's answers are automatically conveyed through the scoring template.

### 5.5. Sample Size

The “sample size formula is calculated as a sample size of students,” as follows:

(1) $$\begin{array}{c} S=A2*\left(c\right)*\frac{\left(1-c\right)}{a2}, \end{array}$$

where *A* = *A* is the value (“1.96 for 95% confidence level”), *P* is the percentage in the decimal value (“.5 used for sample size needed”), *C* is the confidence (for example, “.04 = ± 4”).

### 5.6. Levels of POMS

The POMS test has six different extents of mood swings for more than a period. The POMS test includes “Tension or Anxiety, Anger or Confusion, Vigor, Fatigue, and Depression,” whose division is shown in Figure 4. The POMS test comprises a 5-point scale ranging from “Not at all” to “Extremely,” which is used to estimate their mood states.

It is commonly used for the background of psychotherapy, medicine, and sports science. The POMS and POMS-2 represent the appropriate mechanism to assess mood-related symptoms properly. The POMS and POMS-2 have to cover up independent proportions and somewhat with similar proportions. The study indicates some intersections of the applied instruments concerning psychological well-being.

### 5.7. Total Mood Disturbance (TMD)

Adding up the scores for “Tension, Depression, Anger, Fatigue, and Confusion” minus the score for “Vigor” gives the TMD as follows:

(2) $$\begin{array}{c} \text{TMD }=\;\left(\text{“Tension}+\text{Depression}+\text{Anger}+\text{Fatigue}+\text{Confusion“}\right)‐\text{“Vigor“}. \end{array}$$

### 5.8. Score

• The overall score for “Tension” is calculated by adding up the scores for (Tense, Shaky, On Edge, Panicky, Relaxed, Uneasy, Restless, Nervous, and Anxious).
(i) The overall score for “Depression” is calculated by adding up the scores for (Unhappy, Sorry for things Done, Sad, Blue, Hopeless, Unworthy, Discouraged, Lonely, Miserable, Gloomy, Desperate, Helpless, Worthless, Terrified, and Guilty).
(ii) The overall score for “Anger” is calculated by adding up the scores for (“Anger, Peeved, Grouchy, Spiteful, Annoyed, Resentful, Bitter, Ready to Fight, Rebellious, Deceived, Furious, and Bad Tempered”).
(iii) The overall score for “Fatigue” is calculated by adding the scores (Worn Out, Listless, Fatigued, Exhausted, Sluggish, Weary, and Bushed).
(iv) The overall score for “Confusion” is calculated by adding the score for (Confused, Unable to Concentrate, Muddled, Bewildered, Efficient, Forgetful, and Uncertain about things).
(v) The overall score for “Vigor” is calculated by adding up the scores for (Lively, Active, Energetic, Cheerful, Alert, Full of Peep, Carefree or Vigorous).

The article "Stress-Relieving Video Game and Its Effects: A POMS Case Study" was retracted in 2023. Reasons: unreliable results or conclusions; lack of ethics approval or compliance; missing or withdrawn patient consent; concerns about the data.

### 5.9. Interpreting of POMS-2

In this section, the information applies to interpreting all T-scores presented in this report and interpreting changes in T-scores. Responses on the POMS 2–A are combined to produce a TMD score and scores on six mood clusters: Anger-Hostility (AH), Confusion-Bewilderment (CB), Depression-Dejection (DD), Fatigue-Inertia (FI), Tension-Anxiety (TA), and Vigor-Activity (VA). A scaled score is also calculated for Friendliness (F). TMD is determined by summing the Negative Mood State scales and subtracting VA (a Positive Mood State scale). Friendliness is considered separately as a mood state that may influence the severity of mood disturbance through interpersonal functioning. We evaluated probability-value% and zero-error for the POMS-2 test.

## 6. Results

The survey aims to determine the stress level using a reliable psychological survey paper. The survey collected a variety of information from its participants over six months. A total of 30 participants participated in the survey. The survey asked participants what they felt would be a reasonable explanation for gaming from a menu of items where they could choose more than one answer. This survey allocates the fast evaluation of temporary and changeable emotions as long-term affect states. POMS tests having psychological states can be evaluated rapidly due to the test's ease, which is another noteworthy evaluation feature. The analysis of the participant based on their sex is shown in Table 4.

Table 5 shows the collected data (before and after) from survey statements regarding overall respondents. It clearly shows that the stress level among the respondents has been reduced after gameplay. The analysis data indicate that the video related to reducing stress can be a helpful instrument for quick concern among the participant and reduce the equal level of stress.

### 6.1. Mean

The mean is an arithmetic average of the dataset. The mean is calculated by adding up all the numbers together and dividing by the number of items in the set. The formula for calculating the mean is mentioned in as follows:

(3) $$\begin{array}{c} \mu =\frac{\sum }{N}. \end{array}$$

(3a) $$\begin{array}{c} \left(1\right)\text{ Calculating Mean Before}=\frac{2477}{30}=82, \end{array}$$

(3b) $$\begin{array}{c} \left(2\right)\text{ Calculating Mean After}=\frac{1244}{30}=41. \end{array}$$

Table 6 shows the calculation of mean (Before and after). It offers a clear decline in the TMD in the controlled environment and after playing the game.

The article "Stress-Relieving Video Game and Its Effects: A POMS Case Study" was retracted in 2023. Reasons: unreliable results or conclusions; lack of ethics approval or compliance; missing or withdrawn patient consent; concerns about the data.

Table 7 shows the mean TMD (before and after) and it shows a clear decline in the TMD in the environment and after playing the game.

Figure 5 shows the mean represented graphically to show a clear decline in the TMD in the environment and controlled after playing the game.

### 6.2. Statistical Analysis of Standard Deviation

The standard deviation (SD) in statistical analysis is a measurement of numbers and how it is spread. It is represented by (Greek letter) *σ* symbol. The SD is a statistic measuring the dispersion of the dataset comparative to its mean and is considered the square root of variance. The formula for SD is mentioned as follows:

(4) $$\begin{array}{c} D=\sqrt{\frac{\sum {\left(x-x\right)}^{2}}{n-1}.} \end{array}$$

1. *S* = sample standard deviation.
2. ∑  = sum of total numbers.
3. ∑  = sum of total numbers.
4. $\overset{-}{X}$  = sample mean.

### 6.3. Statistical Analysis of Population Standard Deviation

The population standard deviation is defined as the measure of the spread (variability) of the score regarding the variable. It symbolizes the sum of the “squared” deviations of the scores from their population mean:

(4a) $$\begin{array}{c} \sigma =\sqrt{N\sum x^{2}}-\frac{{\left(\sum x\right)}^{2}}{N^{2}}, \end{array}$$

where*σ* is the population standard deviation, *N* is the size of the population, and X2 means each value from the population.

(4b) $$\begin{array}{c} \text{Standard Deviation}\left(\text{Before}\right)=226,\\ S=\pm 27.71, \end{array}$$

(4c) $$\begin{array}{c} \text{The Population Standard Deviation }\left(\text{After}\right)=\pm 27.25, \end{array}$$

(4d) $$\begin{array}{c} \text{Standard Deviation}=\sum x^{2}=71294,\\ =\sum x^{2}=1547536,\\ \sigma =26.06, \end{array}$$

(4f) $$\begin{array}{c} \text{Population Standard Deviation }\left(\text{After}\right)=\sigma =\frac{\sqrt{N\sum x^{2}}-{\left(\sum x^{2}\right)}^{2}}{N^{2}}\sigma =25.63. \end{array}$$

Table 8 shows the calculation for standard deviation and population standard deviation (before and after). It shows a clear decline in TMD in the environment and controlled after playing the game.

Table 9 shows the mean, standard deviation, and population standard deviation. It clearly shows that TMD has been reduced after playing the game.

### 6.4. Degree of Freedom (*D*f)

The degree of freedom is the self-sufficient value that statistical analysis can estimate and indicates the number of dependent values that vary in an analysis lacking breaking any constraints. Typically, the degree of freedom equals the sample size minus the number of parameters while calculating an analysis. The formula for calculating the degree of freedom is mentioned as follows:

(5) D=fN−1.2,

where *N* is the number of values in the dataset (sample size), calculations of degree of freedom (before + after), and degree of freedom (before, after):

(5a) $$\begin{array}{c} D_{f}=30-1,\\ D_{f}=29. \end{array}$$

The article "Stress-Relieving Video Game and Its Effects: A POMS Case Study" was retracted in 2023. Reasons: unreliable results or conclusions; lack of ethics approval or compliance; missing or withdrawn patient consent; concerns about the data.

### 6.5. Zero-Score

Zero-score is the standard score that provides an idea of mean data, which is far from the mean. But more theoretically, zero-score is defined as the measure of numerous SDs below and above the population mean. To compute Z-score through other data available like the observed value, mean of the sample, and SD, equation (6) denoted the measurement for zero-score.

The zero-score formula is as follows:

(6a) $$\begin{array}{c} Z=x-\frac{\mu }{\sigma }, \end{array}$$

where *Z* is the standard score and *X* is the observed value, mean of the sample. The standard deviation of the sample calculations of zero-score for “before” is as follows:

(6b) $$\begin{array}{c} Z=232.52. \end{array}$$

Zero-score for “after” is as follows:

(6c) $$\begin{array}{c} Z=46.93. \end{array}$$

### 6.6. Probability-Value%

*P*-value% age is defined as the probability of receiving the outcome at least as concentrated as the experimental results of a statistical hypothesis test. *P*-value% is observed by a difference that could have occurred presently by random chance. As a result, the lesser the *p*-value, the larger the statistical inference of the observed difference-value calculation for the Z-table, which is used to calculate the *p*-value. Suppose results in a *p*-value used for a Z-score of negative “1.304.”

Z-table needs to take the positive “1.304” into account, which is the upper right tail. Z-table computes the true *p*-value to obtain a positive *p*-value for a positive Z-score by multiplying with “0.0968,” “2,” and “0.1936.” This would be a *p*-value of 19.36%. *P*-value for a negative Z-score (before) is *Z* = “232.52.” The outcome regarding *p*-value of 01072 and 10.72% for a negative Z-score is 10.72%. For *P*-value for a positive Z-score (before), the outcome regarding the *p*-value of .01072 is multiplied by 2 to get 21.44%. *P*-values (before and after) are in percentage using zero-score. P-value for negative Z-score (after) is Z = 46.93, the results in a p-value of .00003 3%; for a negative Z-score is 3%. The results in a p-value of 3% or 3% are multiplied by 2, to get 6%.

Table 10 shows the overall changes using POMS on different measures, including mean, standard deviation, population standard deviation, Z-score, and *P*-values. It clearly shows the stress level has been reduced to a greater extent. It shows a clear decline in the TMD in the controlled environment and after playing the game.

The article "Stress-Relieving Video Game and Its Effects: A POMS Case Study" was retracted in 2023. Reasons: unreliable results or conclusions; lack of ethics approval or compliance; missing or withdrawn patient consent; concerns about the data.

## 7. Conclusion

This article presented the POMS and POMS-2 used for psychological testing. The POMS and POMS-2 provide understanding effects of games on a person's stress levels and can provide insight into the development and production of games. Different aspects of a person's psychology and reactions are recorded in this scenario. As our game was developed to be a stress releaser, we evaluated stress levels. It was made clear by the survey that our game reduced a certain amount of stress and improved the overall mood of the participants. In future research, we can evaluate the same game through different surveys and methods, like electroencephalography (EEG), which is used to measure brain signals and how they behave concerning stress. Other methods used can also be probed to evaluate stress and how it behaves in our game.

## Figures and Tables

**Figure 1:** POMS strategy.

**Figure 2:** Stress-releasing game.

**Figure 3:** Psychological effects.

**Figure 4:** Pie chart (TMD).

**Figure 5:** Mean graph (before and after).

**Table 1:** world's most stressful countries (2022).

Ranks	Countries
1	Nigeria
2	South Africa
3	El Salvador
4	Mongolia
5	Guatemala
6	Colombia
7	Pakistan
8	Jamaica
9	Macedonia
10	Bolivia

**Table 2:** Stress level in 2021.

Percentage% (%)	Countries
59	Greece
58	Philippines
57	Tanzania
55	Albania
55	Iran
55	Sri Lanka
55	USA
53	Uganda
52	Costa Rica
63	Pakistan

**Table 3:** Stress level in 2020.

Percentage% (%)	Countries
53	Iraq
51	Lebanon
51	Peru
55	Albania
50	Egypt
53	USA
47	Tunisia
46	Iran
76	China
74	Pakistan

**Table 4:** The state of the art in previous studies.

Years	State of the art
2020	Trier Social Stress Test
2020	Perceived Stress Scale
2018	Ardell Wellness Stress Test
2015	Delphi's method
2014	Kessler Perceived Stress Scale
2018	Acceptance and Commitment Therapy (ACT)

**Table 5:** Data collected from survey statements (before and after).

Category	Before (%)	Category	After (%)
Extremely	60	Extremely	20
Fairly	60	Fairly	30
Moderate	80	Moderate	40
A little	40	A little	70
Not at all	20	Not at all	80

**Table 6:** Calculation of mean (before and after).

S.N	Mean (before)	Mean (after) $\mu =\frac{\sum }{N}$
1	62	44
2	132	55
3	105	86
4	100	66
5	101	98
6	84	47
7	124	49
8	133	90
9	76	49
10	102	19
11	95	67
12	44	33
13	94	83
14	74	14
15	121	28
16	76	21
17	102	6
18	91	39
19	104	26
20	78	11
21	62	22
22	36	9
23	40	20
24	29	26
25	63	32
26	67	19
27	79	55
28	61	14
29	89	70
30	53	46
= 2,477/30, *μ* = 82		= 1,244/30, *μ* = 41

**Table 7:** Mean TMD.

Overall POMS changes	Mean
Before	82
After	41

**Table 8:** Calculation of standard deviation (before and after).

	SD (before)		SD (after)	
N	$\overset{-}{X}$	$\overset{-}{X^{2}}$	$\overset{-}{X}$	$\overset{-}{X^{2}}$

1	62	3844	44	1936
2	132	17424	55	3025
3	105	11025	86	7396
4	100	10000	66	4356
5	101	10201	98	9604
6	84	7056	47	2209
7	124	15376	49	2401
8	133	17689	90	8100
9	76	5776	49	2401
10	102	10404	19	361
11	95	9025	67	4489
12	44	1936	33	1089
13	94	8836	83	6889
14	74	5476	14	196
15	121	14641	28	784
16	76	5776	21	441
17	102	10404	6	36
18	91	8281	39	1521
19	104	10816	26	676
20	78	6084	11	121
21	62	3844	22	484
22	36	1296	9	81
23	40	1600	20	400
24	29	841	26	676
25	63	3969	32	1024
26	67	4489	19	361
27	79	6241	55	3025
28	61	3721	14	196
29	89	7921	70	4900
30	53	2809	46	2116
	= (2477) 2 = 6135529	= 226,801, *S* = ±27.71 *σ* = ±27.25	= (1244) 2 = 1547536	= 71294 *S* = ±26.06 *σ* = 25.63

The article "Stress-Relieving Video Game and Its Effects: A POMS Case Study" was retracted in 2023. Reasons: unreliable results or conclusions; lack of ethics approval or compliance; missing or withdrawn patient consent; concerns about the data.

**Table 9:** Calculation of Standard Deviation (Before and after).

Mean	$\mu =\frac{\sum }{N}$	SD	$S\;D={\sqrt{\sum \left(x-\overset{-}{x}\right)}}^{2}/n-1.$	SD population	$\sigma =\sqrt{N\;\sum x^{2}}-\frac{{\left(\sum x\right)}^{2}}{N^{2}}$
Before	82	Before	±27.71	Before	±27.25
After	41	After	±26.06	After	±25.63

**Table 10:** Mean and SD and Population SD (before and after).

POMS overall changes	Mean	Standard deviation (SD)	Population standard deviation (*σ*)	Z-scores (distribution of X)	*P*-values (%)
Before	82	±27.71	±27.25	232.52	21.44
After	41	±26.06	±25.63	46.93	6

## Data Availability

No data were used to support this study.
